This article has been retracted.

# Tumor-Specificity Growth Factor Combined with Tumor Markers in Nuclear Medicine Imaging to Identify Prostate Cancer Osteonosus

**DOI:** 10.1155/2021/7380120

**Published:** 2021-12-10

**Authors:** Xuemin Zhang, Zhengfu Chen

**Affiliations:** Shaanxi University of Chinese Medicine, Clinical Medicine of Chinese and Western Medicine, Hanzhong, Shaanxi 723000, China

## Abstract

**Objective:**

This study has explored the application value of malignant tumor SPE growth factor (TSGF) combined with tumor markers (TM) (TSGF + TM) in nuclear medicine imaging to identify prostate cancer osteonosus (PCO).

**Methods:**

A retrospective analysis for 70 patients with prostate cancer and bone disease admitted to our hospital was performed, 30 healthy persons in the same period were selected as the control group, and the advantages and disadvantages of various examinations were analyzed. All patients were diagnosed with PET whole body bone imaging. Suspicious lesions could be examined by MRI or CT. According to the results of imaging examination, patients were divided into 40 cases of malignant prostate cancer and 30 cases of benign prostate cancer. All the patients underwent ^18^F-FDG-PET imaging, alpha-fetoprotein (AFP), and TSGF + TM determination. The case diagnosis results were compared and analyzed, and the sensitivity (SEN), specificity (SPE), and accuracy (ACC) of various detection methods were calculated. The SEN, SPE, and ACC of positron emission tomography (PET) were 90.9%, 57.8%, and 81.2%, respectively; those of TM were 79.2%, 94.6%, and 69.8%, respectively; and those of TSGF + TM were 95.9%, 100%, and 97.3%, respectively. The accuracy of combined diagnosis of tumors can reach 100%. The AFP and TSGF levels of serum TM were compared and analyzed, and it was found that the benign lesion group and the malignant lesion group showed significant increases compared with the control group, and the difference between the malignant lesion group and the control group was obvious (*P* < 0.05). SGF combined with TM could obtain a more definite diagnosis in PCO.

**Conclusion:**

TSGF + TM combined with ^18^F-FDG-PET imaging showed important clinical value to diagnose the PCO. The imaging accuracy of TSGF + TM combined with 18F-FDG-PET is 97.3%, and the specificity of tumor diagnosis is 100%. Therefore, the TSGF + TM applied in medical imaging and identification of PCO was worthy of clinical promotion.

## 1. Introduction

Worldwide, prostate cancer in developed countries such as Europe and the United States occupies the second place among male malignancies [1]. According to data in the relevant literature, the prevalence of bone loss before treatment in prostate cancer patients is 58%. The prevalence of osteoporosis in these patients was 10%, and the prevalence of osteoporosis after castration was 37%. The incidence of fractures in all patients is 3.4 times that of those without castration treatment, and the incidence of bone metastases in patients with advanced prostate cancer is higher than 80% [2–4]. Prostate cancer is a malignant tumor with the highest incidence among male patients. It has very clear characteristics of osseous metastasis. Among patients with anterior lacrimal gland, 70% of patients suffer from bone metastases [5]. These characteristics will cause the upregulation of the expression of bone formation-related molecules, suggesting that osteoclasts are also involved in the formation of osteoblast metastases. The diagnosis of prostatic bone disease includes the diagnosis of prostate osteoporosis and prostate with bone metastasis [6, 7]. Clinically, there are X-ray bone densitometers and simple tools to predict the fracture risk during the diagnosis of osteoporosis. High-resolution MRI can also provide detailed bone microstructure model images. Castration therapy is very important for the treatment of advanced patients, but castration therapy can cause osteoporosis and increase the risk of fractures and a series of side effects [8].

Tumor specificity growth factor (TSGF) is a collective name for several internationally recognized carbohydrates and metabolites (lipoproteins, enzymes, and amino acids) related to the growth of malignant tumors [9, 10]. TSGH is a special substance produced by malignant tumor cells. During the formation and growth of malignant tumors, it can promote the growth of tumors and the proliferation of surrounding capillaries. It can be released into the blood to reach a certain concentration, all by detecting the level of TSGH in the serum, with great value in the diagnosis of malignant tumors. Tumor-specific growth factor is one of the total multigrowth factors involved in the proliferation of capillaries in and around the tumor tissue during the formation and growth of malignant tumors. It can effectively distinguish cancer from lung cancer, so it can be used for general screening and early diagnosis of malignant tumors [11]. TSGF detection is a very ideal index for clinical detection of malignant tumors. The use of modern biochemical analysis techniques has achieved the purpose of rapid, accurate, and early detection of tumors, and according to the results of clinical reports by relevant experts, the sensitivity (SEN) reached 86% and the specificity (SPE) was above 97% [12, 13]. TSGF shows a strong ability to detect the recurrence of various tumors in the early stage and after treatment, and it has shown a very important effect on the detection of postoperative radiotherapy and chemotherapy. Compared with other tumor markers (TMs), TSGF has a high concentration in the early detection of tumor formation [10]. Medical imaging includes magnetic resonance imaging (MRI), computed tomography (CT), B-ultrasound, and nuclear medicine imaging. With continuous development of the medical industry, nuclear medicine imaging has been widely used [14]. At present, positron emission tomography (PET) and single photon emission CT (SPECT) imaging are the most advanced scanning methods in nuclear medicine imaging. PET imaging and TM detection have shown great clinical value in early diagnosis of cancer, disease progression, treatment response, and judgment of metastasis and recurrence [15, 16]. ^18^F-FDG is a common tracer in clinical practice. It can share the transport protein on the cell membrane with glucose. After the cell membrane, hexokinase is phosphorylated into FDG-6-PO4, so that the metabolism cannot be realized [17] and is retained in the cell to achieve the purpose of imaging. In contrary to other image acquisitions, nuclear medicine imaging of the anatomical results of organs and diseased tissues can form better complete image data [18]. Some researchers have used tumor markers and radionuclide bone imaging results to show that more definite diagnosis results can be obtained, which exerts a role in the staging of the disease.

There are relatively few diagnostic reports about TSGH combined with tumor markers in nuclear medicine imaging to identify prostate cancer. The innovation of this study is that TSGH combined with tumor markers uses nuclear medicine imaging to diagnose and treat prostate cancer patients. This study used TSGF combined with tumor markers to analyze the bone disease of prostate cancer in nuclear medicine imaging. 18F-FDG-PET imaging results were analyzed, TSGF combined with tumor markers were determined, and case diagnosis results were used to perform subsequent comparative analysis, so as to provide a reference for clinical diagnosis and treatment of prostate cancer bone disease.

## 2. Methods

### 2.1. Research Objects

A total of 70 PCO patients from top three hospitals were selected, aged 50–79 (58.56 ± 2.74) years old. 30 healthy persons were selected and served as the control group, aged 51–78 (59.28 ± 2.61) years old. The comparison of general data showed no great difference (*P* > 0.05). All patients underwent the PET whole body bone imaging after diagnosis and magnetic resonance imaging (MRI) or CT examination for suspicious lesions. Based on results of imaging examination, the patients were divided into a malignant lesion group (40 cases) and a benign lesion group (30 cases). And this trial had been endorsed by the Ethics Committee of XXX Orthopedic Hospital. All patients and their families had given informed consent and signed the informed consent forms.

The inclusion criteria were determined as follows: patients who had been in our hospital for a long time, patients who were diagnosed with prostate cancer, patients without history of other malignant tumors, patients without other mental illness, and patients with good understanding and communication skills. The exclusion criteria were determined as follows: patients who disagreed to participate in this study, patients whose clinical data were incomplete, and patients who took long-term oral 5-*α* reductase inhibitors before diagnosis.

All the patients underwent ^18^F-FDG-PET imaging, alpha-fetoprotein (AFP), and TSGF + TM determination. The case diagnosis results were compared and analyzed, and the SEN, SPE, and accuracy (ACC) of various detection methods were calculated.

### 2.2. Tumor SPE Growth Factor

The detection of TSGF could provide an ideal index for the clinic. The TREM1 pathway diagram of TSGF is shown in Figure 1. TSGF has a significant effect on the early diagnosis of malignant tumors and the treatment after recurrence. It is different from other common tumor detection markers. In the early stage of tumor formation, the detection of TSGF has a high concentration in the early stage of tumor formation. In this study, when the subjects were tested for serum tumor markers, each group of researchers took 4 mL of venous blood on an empty stomach and left the upper layer after centrifugation. TSGF used the Roche ELecsys-2010 automatic electrochemiluminescence immunoassay detection, and the colorimetric selection was done by the American Bio Tek ELX808 microplate reader. All operations were carried out in strict accordance with the operating steps in the instructions, and the quality control was also in line with the requirements. TSGF revealed that the cut value was 70U/mL, and if it exceeded the cut value, it was judged as positive.

### 2.3. 18F-FDG PET Imaging

The ECAT EXACT HR + positron emission CT scanner produced by Siemens was adopted for examination (primary collimator half cone angle pseudo 14°). Before the patient underwent the imaging, the medical staff should explain to the patient the details of the examination in advance. Unless there were contraindications, the patient should drink 2–8 glasses of water after the injection of the drug and before the examination. Eating and drinking were forbidden for 6 hours before the examination, urination was required before the examination, and the patient should drink as much water as possible 24 hours after the radiopharmaceutical injection. Some other symptoms of previous patients could also affect the results of bone imaging, such as antibiotics, steroids, chemotherapy, radiotherapy, bisphosphonates, iron therapy, or history of anatomical or functional kidney abnormalities. Prostate-specific antigens in prostate patients can also affect bone imaging. The tracer ^18^F-FDG was used for intravenous injection, and then the patient was instructed to rest for 40 minutes after intravenous injection at 0.15 mCi/kg. The total scanning time was 9 minutes, and the ratio of emission scan to transmission scan time for each bed was 7 : 3. Quantitative analysis was used for nature determination of lesion, and ^18^F-FDG-PET uses the whole body acquisition program and 2D acquisition mode to scan. 2.5 was undertaken as the threshold value; when SUV ≤ 2.5, it was regarded as benign, and when SUV > 2.5, it was regarded as malignant. The images and pictures had two or more senior radiologists for diagnosis and analysis.

### 2.4. Bone Imaging

For early prediction of PCO, adopting corresponding wetness is very important in improving the survival rate and prognosis of patients. 18F-labeled choline is a common tracer in PET imaging of prostate cancer. Bone tissue is composed of inorganic salt, organic matter, and water. The principle of the combination of imaging agent and bone tissue is ion exchange and adsorption. The activity of bone metabolism and local blood flow are factors that affect the uptake of imaging agent by bone tissue [19]. Commonly used bone imaging drugs are 99m Tc-MDP, ^18^F-FDG, and ^18^F–NaF. In this study, ^18^F-FDG-PET was used for scanning with whole body acquisition program and two-dimensional (2D) acquisition mode.  Figure 2 A and B show the images of normal bones, and Figure 2 C and D show the bone imaging results of prostate cancer patients. Compared with normal bone, radioactive accumulation was increased or decreased. The increase or decrease of osteogenic activity can be determined according to the degree of focal accumulation and diffuseness, so as to differentiate and diagnose more complicated lesion distribution, lesion location, and number reduction. Focal radioactive accumulation is reduced, and there is no corresponding increase in radioactive accumulation in the surrounding area of the lesion. This situation is more common in benign lesions. The decrease in the degree of radioactive accumulation and the decrease in the number of lesions indicate that the condition has improved, which may be secondary to local treatment. The increase in the degree of radioactive accumulation and the increase in the number of lesions may indicate disease progression and flash response after treatment. When the soft tissue is observed, it has to pay attention to the abnormal structure of the organ tissue, such as the comparison of the radioactive uptake in the kidney, bladder, and interstitial tissue with normal bone.

### 2.5. Diagnostic Results of Examination Methods

The SEN, SPE, and ACC of each examination methods could be calculated with

(1) $$\begin{array}{c} Sensitivity=\frac{TP}{\left(TP+FN\right)}\times 100\%,\\ Specificity=\frac{TN}{\left(TN+FP\right)}\times 100\%,\\ Accuracy=\frac{\left(TP+TN\right)}{Total}\times 100\%. \end{array}$$

In the above equations, *TP*, *TN*, *FP*, and *FN* referred to the number of true positive cases, true negative cases, false positive cases, and false negative cases, respectively.

### 2.6. Statistical Analysis

The SPSS21.0 software was selected for statistical processing of experimental data in this study. Measurement data conforming to the normal distribution were expressed in the form of mean ± standard deviation ($\overset{¯}{x}$ ± *s*), and those nonconforming were expressed by percentage and frequency (%). The diagnosis result of each method was compared with the diagnosis result of the final gold standard case. The independent sample *t*-test and chi-square test were used for difference comparison. When *P* < 0.05, the difference was statistically significant.

## 3. Results and Discussion

### 3.1. General Data of Patients

After general data of patients were compared, it was found that the differences were not dramatic (*P* > 0.05). As shown in Table 1, the bone metastases of the patients were mainly distributed in the pelvis, clavicle, scapula, and limb bones.

### 3.2. Bone Scanning

Figure 3A shows the concentration of radiation in the lumbar spine and bone scan of a patient aged 53. Figure 3 B shows multiple bone lesions throughout the body, Figure 3 C shows the right bony wing and sacral lesions, and Figure 3 D and E show the local lesions. The red box in the figure indicates the location of the lesion. Bone scan showed high SEN and low SPE for disease diagnosis, so the interpretation of the report should be combined with disease history, physical examination, other examination results, and comparison with previous images. Related technical descriptions include blood flow, blood pool imaging, delayed imaging, injection site, and scanner tomography. The description of imaging agents includes increase or decrease in amount, patterns of abnormal uptake, and structural analysis of bones and soft tissues.

Figure 4 is a medical image of a patient with prostate cancer. It illustrates that the right femoral head showed mixed dense foci under the cortex, the edge of the femoral head was sclerotic, and the inside was cystic, accompanied by abnormal increased radioactive uptake and subchondral bone cyst. The red box in the figure marked the location of the lesion. Figure 44 A presents the position of the prostate. Figure 4 B, C, and D were magnifications of the local lesions in Figure 4 A.

### 3.3. 18F-FDG-PET Imaging

Studies have shown that for the prediction of prostate cancer bone metastasis, the cut-off value of serum bone sialoprotein was 33.26 ng/mL, which was the cut-off value of bone metastasis in patients. ^18^F-FDC is administered by intravenous injection or intravenous catheter, generally 185–370 MBq (5–10 mCi) for adults and 10 mCi for obese patients. Under normal circumstances, ^18^F can be taken up by all bones and then excreted through the urinary system. In the case of renal insufficiency, the ureter and bladder can be visualized. The degree of deposition in the urinary system depends on renal function, water consumption, and the time interval between injection of ^18^F and imaging. With renal insufficiency, radioactive deposits in the urinary system will decrease. The radioactivity in the proximal part of the ureteral obstruction will increase. Chronic severe urine output obstruction can reduce urinary tract radioactive deposition. The radioactive activity of the soft tissue reflects the amount of ^18^F in the blood pool during imaging, which should be reduced to a minimum during imaging. Local hyperemia can cause soft tissue visualization [20]. The uptake of ^18^F in the bones is related to the blood flow of the bones and the formation of new bones. The replacement of the hydroxyl groups in hydroxyapatite by F indicates that the bones are deposited. Since new bone has more binding sites, the uptake of F in the new bone is higher, and the increase in local blood flow will also lead to the uptake of F by the local bone (Figure 5).

Figure 5 shows the imaging results using ^18^F-FDG-PET.

### 3.4. TM Comparison

TMs generally exist in the body fluids, excreta, and tissues of patients. The medical field is constantly evolving, and the detection of tumor markers is also increasing day by day, providing a good breakthrough for the diagnosis of early tumors. After the tumor is formed, the relevant antigens and metabolites will be detected through some biochemical methods or immunochemical quantitative methods. They also have become indicators for early diagnosis of tumors. Tumor markers refer to substances or hosts that are abnormally produced by malignant tumor cells when malignant tumors exist in malignant tumor cells, which can reflect the occurrence and development of tumors and detect tumors for treatment. Common physical examination items include serum carcinoembryonic antigen, biological and chemical methods, and prostate-specific antigens.

At this stage, the medical profession does not have a unified classification standard for TMs, and alpha-fetoprotein (AFP) is also a type of TMs. TSGF is commonly used in the general survey and early diagnosis of malignant tumors, but it has also been increased in the diagnosis of nonmalignant tumors. Research results have shown that this condition may be related to acute inflammation and systemic lupus erythematosus contained in the disease [21]. Boevé et al. (2019) [22] showed that increasing prostate radiotherapy in patients with bone metastases of prostate cancer cannot improve the overall survival rate. In this study, the AFP and TSGF levels of the three groups of serum TMs were compared and analyzed, and the results are shown in Figures 6 and 7. The AFP and TSGF levels in the control group were much lower, showing no obvious difference with the benign lesion group (*P* > 0.05) and remarkable difference with the malignant lesion group (*P* < 0.05).

### 3.5. Comparison of Results of Detection Methods

The results of diagnostic examination methods were analyzed (as shown in Table 2), and it was found that the number of FP detected by the PET + TM was zero; the number of FP detected by the PET was six; the number of TP detected by the PET + TM was 36; the number of FN detected by the PET + TM was 1; the number of FN detected by the PET was 3; the number of TN detected by the PET was 15; and the number of TN detected by the TM was 22.

### 3.6. Comparison of SEN, SPE, and ACC of Detection Methods

Serum TM diagnosis and 18F-FDG-PET imaging are both noninvasive inspection methods, which play very important roles in tumor diagnosis. Choosing an appropriate examination method clinically is very crucial for the determination of examination results and is more accurate. This is more conducive to doctors in adopting more reasonable treatment plans for patients. Compared with traditional imaging technology, PET does not require a collimator, has a higher spatial resolution, and is capable of volume detection. It is a true 3D detection technology. It has a variety of parameters, multiple methods, and the flexibility of multiple radiopharmaceuticals. It is used in physiology. Element tracer is currently an imaging technology that can complete biological display at the molecular level of living organisms [23]. The collection process of PET generally takes a few seconds to a few molecules, and the process of neural activity is calculated in milliseconds, so it cannot quickly reflect the location of neural activity. PET exerts a certain impact on the ACC of the test results under the influence of cardiovascular system.

As illustrated in Figure 8, the SEN, SPE, and ACC of positron emission tomography (PET) were 90.9%, 57.8%, and 81.2%, respectively; those of TM were 79.2%, 94.6%, and 69.8%, respectively; and those of TSGF + TM were 95.9%, 100%, and 97.3%, respectively. The ACC of combined diagnosis of tumors can reach 100%. The sensitivity of PET was significantly higher than that of TM, but the specificity of TM was significantly higher than that of PET, and the accuracy of TM was also significantly higher than that of PET. The specificity of the combined diagnosis of tumors by the two methods could reach 100%. The accuracy of the combined diagnosis of the two methods was significantly higher than that of the TM diagnosis and PET diagnosis alone.

## 4. Conclusion

It was proved in this study that the SEN of ^18^F-FDG-PET imaging was higher in contrast to that of TM, but the SPE of TSGF + TM was 94.6%, which was obviously higher than that of ^18^F-FDG-PET imaging. However, the SPE of the combined application of the two methods reached 100%, the SEN was 95.9%, and the ACC was 97.3%. TSGF + TM can be used in PCO to obtain a more definite diagnosis. TSGF + TM combined with ^18^F-FDG-PET imaging showed important clinical value for clinical diagnosis of PCO, which was worthy of clinical promotion. There were still some shortcomings in this study. (1) The spatial resolution of PET imaging is low, which cannot meet the clinical accurate positioning of anatomy. In actual clinical work, it needs to be combined with other scans such as MRI or CT to show more accurate positioning information so that doctors can make more precise treatment plans. (2) How can the combination of 18F-FDG-PET imaging and TSGF combined with tumor markers achieve 100% sensitivity and accuracy is also an important point of future research.

## Figures and Tables

**Figure 1:** The TREM1 pathway diagram of TSGF (source: http://baike.baidu.com).

**Figure 2:** Comparison of developed pictures. (a, b) Normal bones. (c, d) Prostate patient bones.

**Figure 3:** Bone scanning results of prostate cancer patients.

**Figure 4:** Images of a patient with prostate cancer.

**Figure 5:** Imaging results using ^18^F-FDG-PET.

**Figure 6:** TM level in TSGF. ^*∗*^The difference was statistically obvious (*P* < 0.05).

**Figure 7:** TM level in AFP. ^*∗*^The difference was statistically obvious (*P* < 0.05).

**Figure 8:** Comparison of SEN, SPE, and ACC of three detection methods.

**Table 1:** Comparison of general data of patients.

	Control group	Observation group	*P*
Case	30	70	—
Age (years old)	58.56 ± 2.74	59.28 ± 2.61	2.341
Metastasis	—	12	0.527
Single metastasis	—	8	
≥2 metastases	—	46	0.896
Pelvis	—	28	
Clavicle	—	11	
Shoulder blade	—	18	
Limb bones	—	13	

**Table 2:** Comparison of two detection methods.

Examination methods	Number of TNs (case)	Number of FNs (case)	Number of TPs (case)	Number of FPs (case)
PET	15	3	46	6
TM	22	4	40	4
PET + TM	12	1	36	0
Total	49	8	122	10

## Data Availability

The data underlying the results presented in the study are available within the manuscript.

## References

[1] Smith D. C., Daignault-Newton S., Grivas P. (2020 Aug). Efficacy and effect of cabozantinib on bone metastases in treatment-naive castration-resistant prostate cancer. *Clinical Genitourinary Cancer*.

[2] Litwin M. S., Tan H.-J. (2017 Jun 27). The diagnosis and treatment of prostate cancer. *Journal of the American Medical Association*.

[3] Zhang X. (2019 Nov 21). Interactions between cancer cells and bone microenvironment promote bone metastasis in prostate cancer. *Cancer Communications*.

[4] Ottosson F., Baco E., Lauritzen P. M., Rud E. (2021 May). The prevalence and locations of bone metastases using whole-body MRI in treatment-naïve intermediate- and high-risk prostate cancer. *European Radiology*.

[5] Mayor N., Sathianathen N. J., Buteau J. (2020 Nov). Prostate-specific membrane antigen theranostics in advanced prostate cancer: an evolving option. *BJU International*.

[6] Vale C. L., Fisher D., Kneebone A. (2020 Oct 31). Adjuvant or early salvage radiotherapy for the treatment of localised and locally advanced prostate cancer: a prospectively planned systematic review and meta-analysis of aggregate data. *The Lancet*.

[7] Sawant Dessai A., Palestino Dominguez M., Chen U.-I. (2021 Jan 1). Transcriptional repression of SIRT3 potentiates mitochondrial aconitase activation to drive aggressive prostate cancer to the bone. *Cancer Research*.

[8] Barata P., Agarwal N., Nussenzveig R. (2020 Aug). Clinical activity of pembrolizumab in metastatic prostate cancer with microsatellite instability high (MSI-H) detected by circulating tumor DNA. *Journal for ImmunoTherapy of Cancer*.

[9] Song X., Liang B., Wang C., Shi S. (2020 Aug). Clinical value of color Doppler ultrasound combined with serum CA153, CEA and TSGF detection in the diagnosis of breast cancer. *Experimental and Therapeutic Medicine*.

[10] Tang L., Zhang X.-M. (2020 Jul). Serum TSGF and miR-214 levels in patients with hepatocellular carcinoma and their predictive value for the curative effect of transcatheter arterial chemoembolization. *Annals of Palliative Medicine*.

[11] Zhang Q., Dong G., Wang F., Ding W. (2020). Correlation between the changes of serum COX 2, APE1, VEGF, TGF-*β* and TSGF levels and prognosis in patients with osteosarcoma before and after treatment. *Journal of Cancer Research and Therapeutics*.

[12] Shao T., Huang J., Zheng Z., Wu Q., Liu T., Lv X. (2018). SCCA, TSGF, and the long non-coding RNA AC007271.3 are effective biomarkers for diagnosing oral squamous cell carcinoma. *Cellular Physiology and Biochemistry*.

[13] Yang F., Shi L., Liang T. (2017 Mar 25). Anti-tumor effect of evodiamine by inducing Akt-mediated apoptosis in hepatocellular carcinoma. *Biochemical and Biophysical Research Communications*.

[14] Raju S., Sharma A., Patel C. (2020 Nov). Is there a utility of adding skeletal imaging to 68-Ga-prostate-specific membrane antigen-PET/computed tomography in initial staging of patients with high-risk prostate cancer?. *Nuclear Medicine Communications*.

[15] Ravi Kumar A. S., Lawrentschuk N., Hofman M. S. (2020 Sep). Prostate-specific membrane antigen PET/computed tomography for staging prostate cancer. *Current Opinion in Urology*.

[16] Chen P. C., Liu S. C., Lin T. H. (2021 Mar). Prostate cancer‐secreted CCN3 uses the GSK3*β* and *β*‐catenin pathways to enhance osteogenic factor levels in osteoblasts. *Environmental Toxicology*.

[17] Kyriakopoulos C. E., Heath E. I., Ferrari A. (2020 Nov 1). Exploring spatial-temporal changes in 18F-sodium fluoride PET/CT and circulating tumor cells in metastatic castration-resistant prostate cancer treated with enzalutamide. *Journal of Clinical Oncology*.

[18] Vaz S. C., Oliveira F., Herrmann K., Veit-Haibach P. (2020 Jun). Nuclear medicine and molecular imaging advances in the 21st century. *British Journal of Radiology*.

[19] Smith R. (2020 Jan). Nuclear medicine bone imaging. *Radiologic Technology*.

[20] Beheshti M., Manafi-Farid R., Geinitz H. (2020 Oct). Multiphasic 68Ga-psma PET/CT in the detection of early recurrence in prostate cancer patients with a psa level of less than 1 ng/mL: a prospective study of 135 patients. *Journal of Nuclear Medicine*.

[21] Pianou N. K., Stavrou P. Z., Vlontzou E., Rondogianni P., Exarhos D. N., Datseris I. E. (2019 Jan-Apr). More advantages in detecting bone and soft tissue metastases from prostate cancer using 18F-PSMA PET/CT. *Hellenic Journal of Nuclear Medicine*.

[22] Boevé L. M. S., Hulshof M. C. C. M., Vis A. N. (2019 Mar). Effect on survival of androgen deprivation therapy alone compared to androgen deprivation therapy combined with concurrent radiation therapy to the prostate in patients with primary bone metastatic prostate cancer in a prospective randomised clinical trial: data from the HORRAD trial. *European Urology*.

[23] Vija Racaru L., Sinigaglia M., Kanoun S. (2018 Jul). Fluorine-18-fluorocholine PET/CT parameters predictive for hematological toxicity to radium-223 therapy in castrate-resistant prostate cancer patients with bone metastases. *Nuclear Medicine Communications*.

